RETRACTED

# Clinical Effect of Open Reduction and Internal Fixation for Femoral Neck Fracture in Young Adults and Related Factors of Femoral Head Necrosis

**DOI:** 10.1155/2022/2974830

**Published:** 2022-10-04

**Authors:** Guanghui Lin, Dongliang Yang, Wei Sui

**Affiliations:** Department of Orthopaedics, Xiangyang Central Hospital Affiliated to Hubei University of Arts and Sciences, Xiangyang, Hubei 441021, China

## Abstract

**Objective:**

The purpose of this article is to analyze the clinical effect of open reduction and internal fixation on femoral neck fracture in young adults and to explore the related factors of femoral head necrosis.

**Methods:**

The subjects were young and middle-aged femoral neck fracture patients admitted to our hospital from July 2019 to July 2021. 90 patients were randomly divided into two groups according to different treatment methods. The control group (*n* = 45) was treated with open reduction and internal fixation with hollow nails, while the observation group (*n* = 45) was treated with closed reduction and internal fixation with hollow nails. The clinical effects and adverse reactions of the two groups and the risk factors of avascular necrosis of femoral head were analyzed.

**Results:**

Compared with the control group, the operation time of the observation group was significantly shortened (*P* < 0.05), the amount of bleeding during the operation was significantly reduced (*P* < 0.05), and the incidence of total adverse reactions was significantly reduced (*P* < 0.05). The HSS score and Harris score of the two groups were significantly decreased after treatment (*P* < 0.05), but there was no significant difference in the above scores between the two groups before and after treatment (*P* > 0.05). The related risk factors of necrosis included gender, Garden classification, time from injury to operation, and time of weight bearing after operation (*P* < 0.05) but not related to age and cause of injury (*P* > 0.05).

**Conclusion:**

Open and closed reduction and internal fixation can effectively treat femoral neck fracture in young adults. The risk factors of adverse reactions of osteonecrosis include gender, Garden classification, time from injury to operation, and weight-bearing time after operation.

## 1. Introduction

Femoral neck fractures are common hip traumas caused by transmitted or twisting violence and are primarily fractures caused by rotational and angling stresses from top-down forces acting on the femoral head and neck [1, 2]. The quality of reduction, more than time to surgery, has the most impact on optimizing outcomes and function. There is no consensus in the best fixation construct for these fractures. Neck shortening and varus collapse are the most common challenges of the current fixation options. Use of newer implants is being reported with cautious optimism, and further studies are needed. Young adults are a common population of femoral neck fractures, and the incidence is increasing year by year [3]. At the same time, patients with femoral neck fracture are prone to unhealed fractures and femoral head necrosis, which seriously affects the prognosis of patients [4]. Manipulative reduction and internal fixation are a common clinical treatment for femoral neck fractures, such as open reduction and internal fixation and closed reduction and internal fixation [5]. Fracture internal fixation is aimed at achieving the reduction of the patient's anatomy, restoring the blood supply inside the femoral head, and protecting the femoral head. Especially in young and middle-aged patients, internal fixation has a positive effect on preventing long-term complications such as femoral head necrosis and bone nonunion after fracture surgery [6]. This study analyzed the clinical effect of reduction and internal fixation on the treatment of femoral neck fractures, explored the related factors of femoral head necrosis, and provided reference for clinical treatment.

RETRACTED

## 2. Materials and Methods

### 2.1. Research Objects

The research subjects were young and middle-aged patients with femoral neck fractures admitted to our hospital from July 2019 to July 2021. Inclusion criteria were as follows: age 25–50 years and have typical femoral fracture manifestations. Femoral fractures were diagnosed by CT plain scan combined with three-dimensional reconstruction or magnetic resonance imaging. The clinical data were complete, the patients agreed to this study, and the patients were followed up for more than 6 months. Exclusion criteria were as follows: patients with severe cardiac and renal organic lesions or dysfunction, female patient in pregnancy, patients with severe metabolic system diseases or neurological dysfunction, patients with concurrent malignant tumors, patients complicated with fractures in other parts, and clinical data being incomplete or the subjects dropping out of the study. Ninety patients were randomly divided into two groups according to the treatment method: the control group (*n* = 45) patients were treated with open reduction cannulated screw internal fixation, and the observation group (*n* = 45) patients were treated with closed reduction cannulated screw internal fixation. There were no significant differences in general data such as the gender ratio, age distribution, injury cause, Garden classification, and postoperative weight-bearing time between the two groups (*P* > 0.05). All research subjects were informed and consented, and this study complied with the requirements of the Ethics Committee of Qionghai People's Hospital.

RETRACTED

### 2.2. Methods

90 patients were randomly divided into two groups according to the treatment method: control group (*n* = 45) patients were treated with open reduction cannulated screw internal fixation: supine position, routine disinfection and drape after anesthesia, and Watson-Jones (WJ). A 10 cm longitudinal incision was made through the approach to separate the patient's sartorius muscle and tensor fascia lata muscle space, and the joint capsule of the study object was incised (in a T-shaped manner), and components such as hematoma and loose bodies were removed. The synovium was swollen, and the lateral cortical bone of the upper segment of the femur was exposed, the surrounding contractile muscles were cut off, the fracture site was exposed, the limb was distracted, and the rotation and abduction reduction were performed. After confirming the reduction of the fracture by X-ray fluoroscopy, the guide pin is drilled through the fracture line and then enters the femoral neck. The hollow screw core is used to fix the perspective shot position and the lateral position. First stop bleeding, then wash the joint cavity, suture the joint capsule of the patient, repair the ligament tissue around the joint at the operation site, and finally conduct layered incision. The patients in the observation group (*n* = 45) were fixed with closed reduction cannulated screws: supine position, routine disinfection and drape after anesthesia, traction using a traction bed under “G-arm” fluoroscopy, closed reduction, and “G-arm” fluoroscopy for confirmation; under the reduction and traction to maintain satisfactory reduction, make a small incision on the side of the greater trochanter and drill into the guide needle and take “G-arm” positive and lateral X-ray films and suture the patient's incision after hemostasis.

### 2.3. Observation Indicators

In this study, the clinical effects of the two groups of patients were analyzed, mainly including the operation time, intraoperative blood loss, and hospitalization time. The recovery of the joints of the patients was analyzed, and the changes of the HSS score (HSS knee joint scale) and Harris score (Harris hip function scale) were mainly investigated. This article also analyzes the clinically relevant risk factors for femoral head necrosis, including gender, Garden classification, postoperative weight-bearing time, age, and causes of injury. The Garden classification consists of four grades: type I incomplete stable fracture with impaction in valgus, type II complete but nondisplaced with two groups of trabeculle in line, type III partially displaced with varus with all three trabeculle disturb, and type IV completely displaced with no contact between the fracture fragments.

RETRACTED

### 2.4. Statistical Analysis

SPSS 21.0 software was used for data analysis. The comparison of measurement data between the two groups was carried out first by normality and homogeneity of variance the test, and the comparison of eligible data was analyzed by independent sample *t*-test, and the results were expressed as mean ± standard deviation ($\bar{x}\pm S$). The count data between the two groups were expressed as percentages, and the comparison was performed using the chi-square test. *P* < 0.05 means that there is a statistical difference in the difference.

## 3. Results

### 3.1. Analysis of the Surgical Conditions of the Two Groups of Patients

The study found that compared with the control group, the operation time of the observation group was significantly shortened (*P* < 0.05) and the intraoperative blood loss was significantly reduced (*P* < 0.05), while there was no significant difference in the hospitalization time between the two groups (*P* > 0.05), as shown in Table 1.

### 3.2. Comparison of Postoperative Pain Scores and Hip Joint Function Analysis between the Two Groups of Subjects

The study found that the HSS score and Harris score of the two groups of patients were significantly decreased after treatment (*P* < 0.05), However, there was no significant difference in the scores of the above indicators between the two groups before and after treatment (*P* > 0.05), as shown in Table 2.

### 3.3. Complications

The results showed that the complications of the two groups of subjects mainly included bone nonunion and avascular necrosis of the femoral head and the incidence of total adverse reactions in the control group was significantly higher than that in the observation group (*P* < 0.05), as shown in Table 3.

### 3.4. Analysis of Risk Factors for Femoral Head Necrosis

The study found that the related risk factors of femoral head necrosis included gender, Garden classification, and postoperative weight-bearing time (*P* < 0.05) but were not related to age and cause of injury (*P* > 0.05), as shown in Table 4.

## 4. Discussion

Patients with femoral neck fractures are prone to complications such as nonunion and femoral head ischemia, which have a significant impact on the quality of life of patients. The goal for surgical treatment of femoral neck fractures in young patients is achieving union through an anatomic reduction and stable fixation while avoiding osteonecrosis. The time to surgery remains controversial. At present, manual reduction and internal fixation are usually used in clinical treatment of femoral neck fractures. Manual reduction and internal fixation can effectively achieve the reduction of the anatomical structure, restore the blood supply of the patient's femoral head, and effectively prevent the occurrence of complications. The most descriptive classification used for femoral neck fractures in young patients is the Pauwels classification. As the degree of the femoral neck fracture line relative to the horizontal plane increases, the types differ (<30 degrees type I, between 30 degrees and 50 degrees type II, and >50 degrees type III), Type III fractures are associated with increasing risks of fixation failure, osteonecrosis, and malunion or nonunions. This study found that the operation time, intraoperative blood loss, and incidence of total adverse reactions in the observation group were significantly reduced. The HSS score and Harris score of the two groups of patients were significantly decreased after treatment, but there was no significant difference in the above scores between the two groups before and after treatment. The related risk factors of osteonecrosis included gender, Garden classification, and postoperative weight-bearing time but were not related to age and the cause of injury.

RETRACTED

Fracture internal fixation can achieve the reduction of the anatomical structure of fracture patients and has a positive effect on restoring the normal maintenance of blood in the patient's femoral head. In an analysis of the comparative study of minimally invasive plate fixation reduction surgery with fractures, it was found that the effect of minimally invasive plate fixation reduction surgery was better than that of open reduction and internal fixation and the incidence of complications was lower [7]. The treatment effect of minimally invasive internal fixation on patients with distal tibia fractures is better than that of open reduction and internal fixation with a plate [8], and closed reduction and internal fixation for supracondylar fractures of the humerus have a good surgical effect and can significantly reduce the number of children with family burden [9]. The tibia plateau is an important loading structure of the knee joint, and its fractures are mostly caused by violence directly or indirectly. Tibia plateau fracture is a high-energy trauma, which will have a certain impact on the stability and function of the patient's knee joint, so its treatment has always been a difficult point in clinical treatment. The clinical indicators of the closed reduction group after treatment are better than those of the open reduction group [10], and compared with open reduction, closed reduction and internal fixation can speed up the healing of fractures and promote the recovery of normal physiological function of the knee joint [11]. Previous studies have also confirmed that closed reduction has a very significant effect on the treatment of lower tibial fractures and has a significant effect on the healing rate of fractures with good joint mobility [12] and internal fixation for ankle fractures after treatment has fewer complications and can be significantly improved. For ankle joint function, the effect is significant [13]. This study also found that the operation time of the observation group (closed reduction and internal fixation) was significantly shortened, the intraoperative blood loss was significantly reduced, and the incidence of total adverse reactions was significantly reduced. The HSS scores and Harris scores of the two groups of patients were significantly decreased after treatment, but there was no significant difference in the above scores between the two groups before and after treatment, indicating that open and closed reduction and internal fixation can effectively treat femoral neck fractures in young adults.

RETRACTED

Most intracapsular femoral neck fractures occur in the elderly population. Femoral neck fractures in young patients are much less common and typically a result of a high-energy mechanism. However, femoral head necrosis is a common complication after reduction and internal fixation and its occurrence is related to a variety of internal and external factors [14, 15]. When analyzing the risk factors of femoral head necrosis after internal fixation in elderly patients with femoral neck fracture, it was also found that the time from injury to operation was longer, whether the internal fixator was taken out and the time to take out. The anatomical displacement of the fracture and the effect of reduction after displacement are the clinical risk factors for the occurrence of femoral head necrosis [16]. This study found that the complications of the two groups of subjects mainly included bone nonunion and avascular necrosis of the femoral head and related risk factors for adverse reactions of osteonecrosis included gender, Garden classification, and postoperative weight-bearing time. In future research, we will further carry out the research on the correlation between related risk factors and complications of femoral head necrosis and analyze the correlation coefficient of each factor, so as to provide reference for more reasonable clinical treatment and improvement of patient prognosis.

Therefore, both open and closed reduction and internal fixation can effectively treat femoral neck fractures in young adults and the disease-related risk factors for adverse reactions of osteonecrosis include gender, Garden classification, and postoperative weight-bearing time.

RETRACTED

## Figures and Tables

**Table 1:** Analysis of the surgical conditions of the two groups of patients.

Group		Operation time (min)	Intraoperative bleeding (ml)	Length of hospital stay (d)
Test group	Number of cases (45)	107.53 ± 11.43	54.65 ± 7.86	10.04 ± 2.09
Control group	Number of cases (45)	150.54 ± 12.65	124.56 ± 11.54	11.08 ± 2.15
*t*		4.365	3.980	5.637
*P*		<0.05	<0.05	>0.05

**Table 2:** Comparison of postoperative pain scores and hip joint function of the two groups of subjects.

Group		HSS score	Harris score
Control group (45)	Before treatment	65.87 ± 7.09	45.47 ± 8.43
	After treatment	88.87 ± 9.33	70.54 ± 6.71
*t*		3.895	4.901
*P*		<0.05	<0.05
Test group (45)	Before treatment	66.08 ± 6.71	45.98 ± 8.23
	After treatment	90.54 ± 8.32	72.43 ± 9.06
*t*		5.784	4.413
*P*		<0.05	<0.05

**Table 3:** Analysis of the occurrence of complications.

Group		Does not heal of the bone (%)	Avascular necrosis of the femoral head (%)	Total adverse reaction rate (%)
Control group	Number of cases (45)	11 (12.4%)	2 (2.2%)	13 (14.6%)
Test group	Number of cases (45)	4 (4.4%)	5 (5.5%)	9 (9.9%)
*x*^2^		2.359	4.385	6.995
*P*		<0.05	<0.05	<0.05

**Table 4:** Clinical risk factors for necrosis of the femoral head.

Indexes		Avascular necrosis of the femoral head	Number of cases (35)	Nonavascular necrosis of the femoral head	Number of cases (35)	*x* ^2^	*P*
Gender	Male	25		75		3.524	<0.05
	Female	10		70			
Age	<40 years	15		68		0.458	>0.05
	≥40 years	20		77			
Cause of injury	Hit	20		76		0.771	>0.05
	Fall	15		69			
Garden type	I/II	10		67		3.452	<0.05
	III/IV	25		78			
Postoperative weight-bearing time	<3 months	25		55		3.123	<0.05
	≥3 months	10		90			

## Data Availability

The raw data supporting the conclusion of this article will be available from the authors without undue reservation.
